The article "Effectiveness of Artificial Intelligence Multimedia Courseware in Classroom Teaching Application" was retracted in 2023. Reason: concerns about the peer review.

# Effectiveness of Artificial Intelligence Multimedia Courseware in Classroom Teaching Application

**DOI:** 10.1155/2022/4543875

**Published:** 2022-05-17

**Authors:** Yu Chen, Zhong Chen

**Affiliations:** ^1^School of Economics and Management, Nanchang Normal College of Applied Technology, Nanchang, 330108 Jiangxi, China; ^2^Business School, Xiamen Institute of Technology, Xiamen, 361000 Fujian, China

## Abstract

In the information age, traditional teaching methods can no longer meet the needs of modern students, and the emergence of multimedia courseware teaching mode just solves this problem. Under the trend of education integration, multimedia courseware is becoming more and more important in classroom teaching. Aiming at the characteristics of AI multimedia courseware classroom teaching mode, we discuss the practical application of AI multimedia courseware in classroom teaching and study the classroom teaching mode. Building a distance education platform through network technology can promote the education level. At the same time, the interactive distance education platform serves as a new network platform for system users in the website. In order to speed up the process of education informationization and improve the quality of education, this paper uses .NET technology and video transmission technology to design and implement a multiperson video conversation interactive distance education platform. Through the comparative experiment of two classes in Chengguan Middle School, using this platform for teaching, the average grade of students and the average grade of each course are better than the average grade of nonplatform classes, and the student's cognitive level has improved and is higher than the same level class. The results show that this platform can support a large number of online users and is very good for students of different majors. Through flexible and interactive course interaction, students are more convenient and more independent to learn but also reduce the teacher's time cost and greatly play the advantages of distance education, and the English teaching mode of artificial intelligence multimedia courseware is very popular with students. More than 60% of teachers are satisfied with the teaching mode and above.

## 1. Introduction

With the unremitting efforts of several generations of educators, China has made good progress in information education. Especially in recent years, with the popularity and development of the Internet, various excellent education applications emerge in endlessly. People can obtain corresponding educational resources through more methods or terminals, which greatly improve the fairness of education and make information no longer difficult to obtain, and the overall quality of education has also been significantly improved and has also promoted the process of education reform in China. Among them, the focus is on distance education. Distance education is often referred to as distance learning, a teaching mode for distance learning through the Internet or multimedia guidance. Different from traditional teaching, it can be learned through the Internet and any other means.

At this stage, all major universities in China are basically using traditional teaching methods. Under this traditional teaching method, not only does it cause a lot of financial expenses but it also gradually exposes the drawbacks of lack of flexibility. The cycle of people's knowledge update is also getting shorter and shorter. And because of the dual limitations of traditional education methods in time and space, people in different regions cannot enjoy the same learning opportunities. Scholars and people of different ages have made huge differences in the knowledge structure and cannot make up for it. Because traditional education requires a lot of money, it also causes a considerable number of people to lose the opportunity to receive education and so on. In this ever-evolving society, knowledge becomes more and more important, and the burden on schools will become heavier. The burden of schools will become heavier and heavier. It can be said that traditional teaching methods are no longer sufficient and difficult to adapt to the needs of modern society.

With the continuous development of technology, the need for knowledge is growing. How to make teaching and training meet the different needs of different people at different times and at different times is an issue that needs to be considered in today's society. The network is developing rapidly, and the information technology field has undergone earthshaking changes. Therefore, in this context, the development and design of the distance education platform began. The distance education platform has unique advantages in teaching because of its huge amount of information and flexible interaction with students. The distance education platform can maximize the subjective and independent learning of students without a fixed location and time constraints. From the previous centralized and unified education mode to the flexible and flexible education mode for students, it also serves many people who have not entered traditional colleges and universities for various reasons and provides them with the opportunity to receive education flexibly, thus making education more social.

However, with a variety of excellent network education applications emerge in endlessly, distance education has become very common, which has also brought new problems. More distance education platforms can only stay in the classroom education and transfer to the Internet. The advantages of distance education are not well reflected, and most distance education courses are small-scale courses of college-specific majors and their audiences also limited to students in specific majors. At the same time, many courses lack teacher-student interaction and are boring and greatly reduce the advantages of the distance education platform. Modern distance education is mostly achieved through websites. Nowadays, many domestic and foreign companies have researched and developed many web-based distance education systems, mainly including distance education platforms based on ASP, PHP, JSP, and other technologies, including network colleges and virtual universities. Nowadays, the distance education team is constantly growing, and the development of interactive distance education platform is getting more and more attention from the society.

## 2. Literature Discussion

The rapid popularity and application of the Internet around the world have made it possible for humans to share related resource space. These conveniences are specifically described in the literature [1]. Among them, .NET technology has played a huge role. In order to realize the remote monitoring and intelligent management of the litchi garden environment, Yu et al. [2] designed a remote monitoring system for intelligent irrigation of Lizhiyuan based on http://ASP.NET/ technology. Use ASP.NET technology to display the environmental parameters of litchi garden in real time. The user can grasp the soil environment information of litchi garden, the residual energy of each node, control the irrigation status, and learn the lychee planting knowledge through real-time monitoring of the litchi garden environment and make intelligent irrigation decisions in time. Honglei and Liu [3] developed a stadium asset management system based on .NET technology. It is easier to implement more complex solutions based on .NET technology, which can better improve the efficiency of stadium asset management and reduce asset management risks. Jinjin and Chen [4], for the deficiencies in PE teaching, combined with .NET technology, optimize the development based on .NET Technology. The results confirmed that the design and development of the sports selection system based on .NET technology not only satisfies the students' demand for sports electives but also improves the utilization efficiency of sports elective resources, increases 34.0%, and exerts positive design and development benefits. Wei [5] constructed a quality and safety traceability system for fresh agricultural products based on the characteristics of fresh agricultural products and system development needs, using .NET technology, bar code technology, and database technology. The realization of this system is of great significance to improve production management and information sharing and guarantee the quality and safety of fresh produce. Sun [6] designed and developed the aerobics teaching website based on .NET technology. The teacher can publish the shared teaching resources on the aerobics teaching website, arrange the viewing of student homework, realize the independent online communication between the students and the teacher, and improve the application performance of the aerobics teaching website.

Video conversation is a way of communication that allows participants to communicate in an immersive way, which brings the distance between people in different regions who have communication needs [7], for example, a more typical representative, video conferencing [8]. It not only brings people a convenient meeting mode but also provides people with more services to ensure that users can easily make video conference calls online. Hu and Feng [9] designed a remote monitoring system for power grids to improve the level of environmental pollution control. The system has good real-time video transmission, high definition, low monitoring energy consumption, and high monitoring accuracy, which can greatly help environmental pollution control. Wei [10] designed a multimedia video conferencing system, pointing out that the video call function and multiparty video resource sharing function break the geographical restrictions on information. Guo et al. [11] studied the scene-experienced social games dominated by multiperson audio and video technology and found that the constructed ultra-real social experience has made its real-world influence increasingly enhanced and even has a plastic effect on the potential future of human beings. Zheng and Yuting [12] found that classroom video analysis provides new methods and techniques for obtaining data and improving the empirical level of research for the research teaching and learning process and its related causes. Yuanhang and Yanguang [13] designed and implemented a SIP-based video call system and established and managed a video call session through the SIP protocol, which has certain practical significance in the field of intelligent communication and life entertainment.

Due to the advantages of distance education, traditional teaching can be effectively supplemented, and the effect of teaching can be improved. Many research teams have introduced interactive distance education platform into teaching, so that the status quo of education informationization can be quickly changed. European and American countries have started earlier in distance education. Since the rapid development of teaching television in the 1950s and the development of social science research after the Second World War, distance education has always been a favorite of educational researchers compared with so-called face-to-face education [14]. In the 1960s, Schramm and Oberholtzer conducted a study comparing teaching television (ITV) with classroom instruction [15]. In addition, Schramm summarizes the results of more than 400 scientific design and statistical processing of ITV and classroom teaching comparisons. He concluded the following: “We can confidently say that students can learn from them and they can learn quickly and effectively.” The specific performance is that many foreign governments have included the construction of distance education platforms in the budget for infrastructure construction, including the US Department of Education's GEM project and the virtual education network established by each state in Australia [16]. One-third of universities in the United States allow students to obtain degrees through online education [17]. In the early 20th century, the United Kingdom had a nationwide education network, which enabled schools across the country to connect via the Internet and distribute e-mail addresses to all students, providing convenience and policy support for the popularization of distance education [18].

China's long-distance education started relatively late. It was not until 1994 that the country carried out the first national demonstration project-educational research network [19]. Although it started late, China unanimously believes that distance education has good prospects; so, it has been actively investing money, manpower, and material resources since its development. By 2018, 68 universities across the country have been approved to open distance education [20], which has broadened the space for higher education in China and provided educational opportunities for those who cannot enter ordinary higher education institutions for various reasons. It also built a platform for learning for our citizens to receive lifelong education. Xin [21] studied the application of virtual reality technology in the distance education platform and the implementation of VRMDEP, proposed the overall framework of building VRMDEP, designed the virtual synchronous and asynchronous teaching system, and built the simulation scene to realize the interaction between users. This is a distance education platform that combines virtual reality technology. It can use 3D modeling technology to build virtual classrooms and classrooms, so that learners can be in the real classroom and realize human-computer interaction, which will help enhance the real experience, enhance the fun of learning, and let more people feel the campus life. To effectively address people's needs to learn anytime and anywhere, Huang [22] proposed a mobile intelligent education platform based on wireless network technology and mobile intelligent mobile terminal technology, which enables students to participate in learning activities more passionately and effectively improve teaching efficiency. China Cardiovascular Health Alliance [23] introduced a distance education platform in the field of tea culture. Through the distance education platform, the connotation and display form of the baptism tea culture that has gone through thousands of years is gradually expanding and extending, so that the tea culture can be inherited and spread. In the medical field, the distance education platform has also contributed. The 20 hospitals of the China Cardiovascular Health Alliance conducted a “face-to-face” difficult case consultation through the Chinese distance education platform to give the best treatment plan [24, 25]. This enables the grassroots doctors to learn and communicate with the top experts in cardiovascular disease in China without leaving the department, thereby strengthening the ability and technical level of the primary doctors, thereby increasing people's trust in the grassroots doctors, and gradually achieving graded diagnosis and two-way transfer diagnosis [26, 27].

This paper provides a development suggestion for the improvement and improvement of course teaching under the information education and can also provide new ideas for the research in the field of distance education interactive platform.

## 3. Design of Interactive Distance Education Platform for Multiplayer Video Conversation Based on .NET Technology

### 3.1. Key Technologies

#### 3.1.1. B/S Architecture

The development of this platform uses the B/S architecture. The B/S architecture refers to the browser server architecture, which is called browser/server. Browser refers to the browser in the user's computer. Compared to the C/S (client/server) architecture, the B/S architecture does not need to be installed, just use the browser that comes with the computer. In the B/S architecture, the web browser is responsible for simple logic and display logic, while the rest of the processing logic is done by the web server. The B/S mode can be applied to the WAN, with strong interactivity and wide application range.

#### 3.1.2. .NET Framework

One of the biggest conveniences of the .NET framework is that it can communicate on the server, which has further innovations at the language level. The basic structure is shown in Figure 1. .NET is composed of two important components: the common language runtime (CLR) and the .NET framework class library (FCL).

The CLR is the operating environment of the framework. In a sense, the CLR has similar features and principles to Java. Its main responsibility is to sequence and maintain the program code written by the developer, including memory management, thread execution, code execution, code full verification, and compilation.

FCL is a public base class library for the .NET framework. This library provides many object-oriented classes for all .NET programs. Classes can provide a series of complex functions such as data manipulation, string manipulation, and database connection. One can also use these classes to efficiently write such applications.

#### 3.1.3. Video Technology

The development of this platform uses the MPEG-4 video coding standard. MPEG-4 is a solution developed by the International Organization for Standardization for multimedia communications, from simply improving compression efficiency to developing a universal content-based multimedia coding standard. Its main feature is to encode the content in the image. The specific encoding object is the audio and video in the image, which is called AV object. MPEG-4 is built around the encoding, storage, transmission, and combination of AV objects. Compared with the previous multimedia coding standards MPEG-1, MPEG-2, H.261, and H.263, MPEG-4 can provide higher compression efficiency due to the adoption of a new compression algorithm such as zero-wavelet transform. It is structurally adaptable and scalable, adapts to the rapid development of software and hardware, incorporates new technologies in time, allows flexible allocation of code rates between different objects, allocates more bytes to important objects, and allocates fewer bytes to secondary objects, which may result in better results at lower bit rates. Natural and synthetic video and audio objects can be easily integrated.

Since the current Internet cannot provide any QOS guarantees, MPEG-4 faces many difficulties in the real-time transmission of video, which are summarized as follows: bandwidth limitation, delay, and data loss and errors in transmission. We need to make correct estimates and then pass the rate control to make the output code stream meet. The optimality of a certain evaluation index is achieved under the condition of bandwidth limitation. The specific practices are as follows:

1. Bandwidth estimation: feedback congestion control can be implemented by RTP and RTCP on top of the UDP protocol. The loss of the current network transmission data of the receiving end is counted, the packet loss rate is fed back to the transmitting end, and the transmitting end adjusts the estimation of the bandwidth used by the current network by the loss rate. (2) Rate allocation: in order to obtain optimal video quality, bandwidth resources need to be allocated reasonably between different frames, video objects, and even macroblocks. In fact, considering that the human visual system is far more sensitive to low-frequency information than high-frequency information, the source stream can be low-pass filtered with a Gaussian filter and then encoded with a specific algorithm, which can be reduced by sacrificing the peak signal-to-noise ratio (PSNR). The boundary effect of macroblocks achieves the integrity of real-time video transmission and provides quality assurance for multiperson video sessions

#### 3.1.4. Database Access Technology-ADO.NET Technology

ADO.NET is a set of object-oriented libraries for interacting with data sources. It is created for the .NET framework. It provides consistent access to data sources such as Microsoft SQLserver, Oracle, and data sources exposed through OLE DB and XML. Applications can use ADO.NET to connect to these data sources and retrieve, manipulate, and update data. The architecture of ADO.NET is shown in Figure 2.

The purpose of designing ADO.NET is to help developers use efficient multitier database applications on the Internet, and the ADO.NET object model provides such a means. The ADO.NET object model is shown in Figure 3.

In Figure 3, the class that contains the ADO.NET object model is shown. The dotted line in the middle divides the object model into two parts. The object to the left of the dashed line is the connection object. These objects communicate directly with the database to manage connections and transactions, as well as retrieve data from the database and submit changes to the database. The object to the right of the dashed line is a nonconnected object that allows the user to process the data offline.

### 3.2. Platform Function Module Division

The educational platform for multiperson video conversation based on .NET technology mainly includes five functional modules, as shown in Figure 4.

The user management module is mainly for users who manage different roles. The course management module mainly includes functions such as course release, course announcement management, and course description management.

The video management module mainly includes multiparty video session management, multiparty video session recording and playback, and question and answer problem management.

The online evaluation management function module mainly includes the addition of the examination questions, the setting of the examination answers, the given scores of the examination questions, and the score statistics function of the whole evaluation.

The resource management module is mainly for uploading, downloading, playing, viewing, and deleting resources such as course videos, course PPT, and course lectures of the distance education platform.

## 4. Implementation of Interactive Distance Education Platform for Multiplayer Video Conversation Based on .NET Technology

This section is designed and implemented according to the designed functional modules. The interface of the distance education platform is shown below.

### 4.1. Platform Main Interface

The main interface of the platform is shown in Figure 5. The overall design of the interface follows the principle of simplicity.

By clicking on the left navigation bar, users can enter the corresponding interface of user management, course management, video management, online testing, and course resources. You can see the teacher's wonderful lecture video in the “Lecture Hall.” In order to facilitate students to inquire about the curriculum, there is a corresponding menu entry in the home page. In the “Latest Online” section, users can see the learning resources provided by the distance education platform in the near future after clicking the picture. “Learning Dynamics” shows some of the platform's results and various types of learning information. Users can get more learning dynamic information by clicking the “View More” button.

### 4.2. Video Classroom Interface

The teacher lectures in front of the dedicated camera equipment, and the student can listen to the teacher's class content through the personal terminal. On the student's personal terminal, the teacher's real-time dynamics will be played, and the effect is shown in Figure 6.

When students need to communicate with the class teacher, they can click the “Join Video Session” button at the bottom of the screen to enable a real-time interactive video session for multiple people after the teacher allows. When you want to end your session, just click the “Exit Video Session” button. The whole process is very convenient. The distance education platform gives teachers certain permissions, including whether to allow students to enter multiperson interactive video sessions. This permission helps teachers maintain classroom order at the remote end so that students do not interfere with each other.

### 4.3. Online Test Interface

The online test questions cover many subjects such as language, mathematics, English, and physics. Here is an example of a mathematical test interface, as shown in Figure 7.

As shown in Figure 7, the online test interface includes the topic of the test topic, the type of the topic (multichoice questions, multiple-choice questions, fill-in-the-blank questions, application questions), the number of participants, and the correct rate of answering questions.

### 4.4. Course Resource Interface

Click “Course Resources” on the distance education platform to enter the interface is shown in Figure 8.

In the “Course Resources Interface,” users can see the course resources of different contents in different disciplines, and click on the corresponding module to enter the course resource detail page. At the same time, the user clicks the “Previous” and “Next” buttons in the lower right corner of the page to perform page turning operations to view more course resources; click the “Back” button to return to the main interface of the distance education platform.

## 5. Comparison of Effects

In order to explore the practical application of the multiperson video dialogue interactive distance education platform based on .NET technology in this article, the use of the distance education platform by teachers and students of a high school is calculated. Understand students' learning in the distance education platform (test scores and cognitive level). The participating students are the class of distance education platform of Chengguan Middle School (hereinafter referred to as class 1) and the class of nondistance education platform of the same level (hereinafter referred to as class 2). The participating teachers are all teachers in various disciplines, and their subjects include the following six: language, mathematics, English, physics, chemistry, and biology.

### 5.1. Comparison of the Performance of Two Classes in Different Teaching Modes

1. The average scores of the total scores of the whole class and the average scores of each subject in the final exams of senior one are shown in Figure 9
2. The average scores of the total scores of the classes and the average scores of each subject in the final exam of senior two are shown in Figure 10
3. The average scores of the total scores of the classes and the average scores of each subject in the final exam of senior three are shown in Figure 11

Through comparison, we can clearly know the following:

1. The average score of the experimental class is higher than that of the students of the same level in the control class
2. The average scores of the students in the distance education platform class are basically the same as those of the nondistance education platform class at the same level. But as time went by, the gap between the two classes of students gradually emerged. Among them, the vast majority of students in the distance education platform class have achieved very good results in subjects considered difficult to learn, such as mathematics and physics. This undoubtedly shows that the teaching mode of the interactive distance education platform is still significantly better than the traditional teaching mode in the physical classroom and has a better teaching effect
3. The language subjects that are deeply loved by students are basically equivalent to the nondistance education platform classes of the same level. This shows that in the subject of Chinese language treatment, only when the accumulation of long-term cultural knowledge is strengthened, the language level of students can be truly improved. At the same time, it also reflects the study of the language subject. It is not enough to rely on only a few minutes of study in the classroom

### 5.2. A Comparative Analysis of the Cognitive Level of Distance Education Class Students and Class Students of the Same Level of Nondistance Education Platform

The student's cognitive level is reflected in the test paper. Take the chemical test paper as an example to analyze the student's test papers. The questions in the chemistry paper include multiple-choice questions, fill-in-the-blank questions, and answer questions. Different topics of the test paper are scientifically divided into different cognitive levels. Cognitive levels are divided into three categories, namely, level of understanding, level of understanding, and level of application.  Table 1 is a comparison of the cognitive level of the students in the distance education platform class and the students in the same level nondistance education platform class under the two teaching modes.

As shown in Table 1, the scores of students studying on the distance education platform in terms of comprehension level questions, understanding level questions, and application level questions are differently higher than those of nondistance education platform class students. Among them, the gap of average scores of comprehension level questions is the biggest. Further analysis of the reasons can be found: the students in these two classes have different attitudes towards learning. For example, when they encounter learning problems, most of the students in the distance education platform class first react to thinking by themselves to solve problems. If they cannot solve the problem, they will turn to teachers or other students who have better academic performance through multiperson level conversation function on the distance education platform. In contrast, this is rare among nondistance education platform class students at the same level. In the long run, the learning effect of students in distance education platform classes has been significantly improved, and students in nondistance education platform classes at the same level are far behind.

### 5.3. Teachers' Satisfaction with Classroom Order, Atmosphere, Interaction, and Teaching Effects Is Shown in Figure 12

From the survey of classroom order in Figure 12, we can see that teachers are very optimistic about the classroom order of interactive distance education platform. 62% of teachers think that the classroom order is “good,” 37% of teachers think that the classroom order is “general,” and only 1% of teachers think that the classroom order is “very bad” [28, 29].

The survey of classroom atmosphere shows that the situation is not very optimistic. 64% of teachers hold a “general” attitude in the classroom atmosphere survey of distance education platform. 15% of teachers feel that the classroom atmosphere is not active enough and a little “lifeless.” The ratio of the two is as high as 79%. The reason is that most teachers who teach on the distance education platform think that their students feel that they are “visitors” of the distance education platform. A small number of teachers are basically language teachers [30, 31]. This platform is a multiperson video conversation interactive distance education platform based on .NET technology. Teachers also do not use the function of multiperson video conversations in different degrees during the class [32].

In an interactive satisfaction survey, 17% of teachers have a “satisfied” attitude, 59% of teachers have a “general” attitude, which together account for 76%, and the overall situation is still optimistic. Because the distance education platform mentioned in this paper is different from the traditional live broadcast education platform, on the previous live broadcast type education platform, when the lecturer lectures, the students cannot communicate with the teacher in real time, and the teacher cannot see the students' expression. In the distance education platform of this article, teachers and students can explore through the interactive mode of multiperson conversations. Teachers can know the situation of students in time and correct their progress in real time [33].

In the survey of the teaching effect of the distance education platform, the results showed that the number of people who were “very satisfied” was 33%, those who were “satisfied” were 31%, and those who held “general” attitudes were “26%.” The results of the survey are also generally optimistic.

In general, in the eyes of teachers, the interactive distance education platform is generally better than the traditional teaching method, which is mainly reflected in the following: ① students in the distance education platform class can get more excellent teaching resources than the students in the nondistance education platform class. However, if students want to master these teaching contents, they often need to spend more energy to solve the unintelligible knowledge in the classroom. They will invest a lot of time in after-school review, prestudy, and exercise training. The traditional students who teach mathematics mode pay more attention to the questioning of teachers and do not want to solve themselves independently. Over time, students in the distance education platform class can learn anytime and anywhere, their thinking is more open, and they will develop the habit of active learning more naturally. ② In the classroom of traditional education, students have many methods and learning skills to solve problems. Coupled with the guidance of the remote tutor, the students in the distance education platform class will express their opinions more easily and reasonably in the classroom, using different methods to solve the problem raised by the teacher. Therefore, students in the distance education platform class are more independent in solving problems than students in the same level nondistance education platform class. ③ The distance learning mode of the distance learning mode is more obviously caused by many factors. The time for teachers to teach is also limited. It is still impossible to form a one-to-one teaching mode. Therefore, as long as the remote students do not understand the meaning of the front-end teacher, it is difficult to interact with the front-end teacher in real time or only get a part of the teacher's instructions. In order to learn properly, our remote students will think of ways to improve their abilities after class. Therefore, when comparing the comprehension level test, the average understanding ability of the students in the distance education platform class will be significantly higher than that of the nondistance education platform class in the same level. At the same time, in the investigation, it is not excluded that students do not follow the classroom discipline of the distance education platform, go to sleep in class, and do not want to learn after class.

## 6. Conclusion

The application of artificial intelligence multimedia technology has changed the traditional teaching methods, strengthened the teaching methods, improved the teaching mode and the effect, and expanded the scope of students' knowledge. This research investigates the current situation of AI multimedia courseware-assisted teaching and understands the teachers' attitude towards multimedia courseware in classroom teaching. At the same time, through the questionnaire survey, classroom observation, and interview, we found that multimedia courseware in classroom teaching, the results show that multimedia courseware teaching is generally popular today and pay attention to personalized learning and independent learning, conducive to the improvement of students' learning effect, and teachers can also effectively help students improve the comprehensive learning ability. In response to the current urgent needs of the people and shortcomings of the domestic distance education platform, this paper designs and develops a distance education platform. The main work of the paper is summarized as follows:

1. According to the status quo of distance education, an interactive distance education platform based on multiperson video conversation is proposed
2. Most distance education platforms generally adopt the C/S mode. Maintenance and upgrade are more troublesome, and the client is burdened with a third-party plug-in. The platform was developed using .NET technology, web technology, video technology, etc.
3. Verify the effectiveness of the platform. After using the platform, students' scores have improved

Although this paper has conducted in-depth research on course teaching using the distance education platform, there are still many deficiencies, and my academic level research is also limited. Teaching methods and means continuously improves the quality of teaching.

## Figures and Tables

**Figure 1:** The basic structure of the .NET framework.

**Figure 2:** ADO.NET architecture.

**Figure 3:** ADO.NET object model.

**Figure 4:** Division of overall functional modules.

**Figure 5:** The main interface of the distance education platform.

**Figure 6:** Video interface.

**Figure 7:** Math online test interface.

**Figure 8:** Course resource interface.

**Figure 9:** The average scores of the whole class and the subjects in the final exam of senior one.

**Figure 10:** The average scores of the whole class and the subjects in the final exam of senior two.

**Figure 11:** The average scores of the whole class and the subjects in the final exam of senior three.

**Figure 12:** Comparison of teacher satisfaction survey results.

**Table 1:** Cognitive level comparison analysis table.

Class	Average score of understanding level	Average score of comprehension level	Average score of application level
Class 1	16	23	31
Class 2	13	16.5	26.3

## Data Availability

The data that support the findings of this study are available from the corresponding author upon reasonable request.
